# Effects of activating GABAB1 receptor on proliferation, migration, invasion and epithelial-mesenchymal transition of ovarian cancer cells

**DOI:** 10.1186/s13048-020-00726-4

**Published:** 2020-10-24

**Authors:** Jun Gao, Yao Gao, Shixin Lin, Xia Zou, Yukai Zhu, Xintong Chen, Hong Wan, Hong Zhu

**Affiliations:** 1 Department of Obstetrics and Gynecology, the Third Affiliated Hospital of Nanchang University, Xiangshanbei Road 128, Donghu District, Nanchang, 330008 Jiangxi China; 2 Postgraduate Department, Jiangxi Medical College of Nanchang University, Nanchang, 330008 Jiangxi China

**Keywords:** GABAB1 receptor, Ovarian cancer, Epithelial-mesenchymal transition, Baclofen, G protein-coupled receptor

## Abstract

**Objective:**

This study aimed to explore the effects of activating GABAB1 receptor by baclofen on proliferation, migration, invasion and epithelial-mesenchymal transition (EMT) of ovarian cancer cells.

**Results:**

One hundred μmol/L, 200 μmol/L and 300 μmol/L were selected as low, medium and high baclofen concentrations respectively. Cells were divided into four groups: Control, 100 μmol/L, 200 μmol/L and 300 μmol/L. Compared with the control group, the viability, colony formation, migration and invasion of SKOV3 cells were inhibited, and the apoptosis of SKOV3 cells were enhanced significantly at 200 μmol/L and 300 μmol/L baclofen. Moreover, they changed significantly with the increase of baclofen concentration. Compared with the control group, the expression of E-cadherin and GABAB1 increased and the N-cadherin expression decreased significantly in 200 μmol/L and 300 μmol/L groups. Higher concentration of baclofen induced higher expression of E-cadherin and lower expression of N-cadherin.

**Conclusion:**

Baclofen inhibited the proliferation, cloning, migration, invasion and EMT of ovarian cancer cells by activating GABAB1 receptor. These results might contribute a lot to clarify the role and possible mechanism of GABAB1 receptor in ovarian cancer.

## Background

Ovarian cancer is the third most common malignant tumor in female reproductive system, and it has the highest mortality rate among gynecological tumors [1]. Ovarian cancer is featured with hidden onset, difficulty in early detection, high degree of malignancy and easy recurrence and metastasis [1]. Ovarian cancer not only seriously harms the patients’ psychological and physical health, but also imposes a heavy financial burden on the patients and society.

Epithelial tumors are the most common among all primary ovarian cancer, accounting for about 50–70% [2]. Due to the low response rate to drug therapy and poor prognosis, the mortality rate of epithelial ovarian cancer is still high [3–5]. Intensive study of epithelial ovarian cancer is of great economic and social significance for the early detection and treatment of ovarian cancer. The development and progression of ovarian cancer is a multi-factor and complex process, where multi-gene and multi-signal pathways are involved. Its specific pathogenesis has not yet been fully understood. However, the proliferation, migration and epithelial-mesenchymal transition (EMT) of tumor cells are undoubtedly important factors for the development and invasion of epithelial ovarian cancer [6].

G protein-coupled receptor (GPCR) is considered to be a successful source of drug targets. The targets of over 50% of clinical drugs and drugs under development are GPCRs, and nine Nobel Prizes have been awarded for the important discoveries in the field of GPCR [7]. γ-aminobutyric acid (GABA) is an inhibitory neurotransmitter and it is the main neurotransmitter in the central nervous system. It plays a crucial role in regulating the excitability of nerve cells [8]. The execution of GABA function is inseparable from its unique receptor system. Receptors of GABA include ionic receptors such as GABAA and GABAC and metabolic receptor GABAB [9]. GABAB receptor regulates downstream activities through G protein coupling, such as inhibiting adenylate cyclase, activating potassium channels, and inhibiting voltage-dependent calcium channels, and it also play an important role in the development process [10–12]. Neurotransmitters are found to play an important role in the regulation of tumor cells through affecting the growth and development of tumors [13]. GABA inhibits the growth of lung cancer cells through GABAB receptor [14]. For patients with ovarian cancer, increased levels of GABA in urine represent a worsening of the cancer [15]. The expression of GABAB receptor may be closely related to the growth of cancer cells. As a member of the GPCR family, GABAB1 receptor participates in many important physiological activities such as the generation of learning and memory and the transmission of synaptic signals. The over-activation or inhibition of GABAB1 receptor will cause various neurological disorders [16]. GABA is a natural ligand of GABAB1 receptor and GABAB1 is the most active subtype of GABAB [9]. Naumenko et al. report in 2017 that baclofen has two stable coupling sites with GABAB1, which is a specific agonist of GABAB1 receptor [17].

Therefore, in this study, we aimed to explore the effects of activating GABAB1 receptor by baclofen on the proliferation, migration, invasion and EMT of SKOV3 cells, so as to clarify the role and possible mechanism of GABAB1 receptor in ovarian cancer. Human ovarian cancer cell line SKOV3 was taken as the research object for its extensive use as a model cell line in ovarian cancer research. This study might provide a theoretical basis for the further development of anti-cancer drugs coupled with GABAB1 receptor.

## Materials and methods

### Materials and cells

Baclofen (HY-B0007/CS-2990) was purchased from MedChemExpress (Monmouth Junction, NJ, USA). CCK-8 kit was provided by Keygen Biotech (Jiangsu, China). Annexin V-fluorescein isothiocyanate (FITC)/propidium iodide (PI) apoptosis kit was gotten from Multi Sciences (Zhejiang, China). Trizon Reagent, Ultrapure RNA extraction kit, HiFiScript cDNA synthesis kit and UltraSYBR Mixture were bought from CWBIO (Beijing, China). RIPA buffer was provided by Applygen (Beijing, China). Mouse anti-glyceraldehyde-3-phosphate dehydrogenase (GAPDH) monoclonal antibody (TA-08), peroxidase-conjugated goat anti-rabbit IgG(H + L) (ZB-2301) and peroxidase-conjugated goat anti-mouse IgG(H + L) (ZB-2305) were obtained from ZSGB-BIO (Beijing, China). Rabbit anti-E-cadherin monoclonal antibody (ab407742), rabbit anti-N-cadherin polyclonal antibody (ab18203) and mouse anti-GABAB1 receptor monoclonal antibody (ab55051) were purchased from Abcam (Cambridge, MA, USA).

Human ovarian cancer cell line SKOV3 (BNCC310551) and human normal ovarian cell line IOSE80 (BNCC340318) were obtained from BeNa Culture Collection (Beijing, China). The cells were cultured in McCoy’s 5A medium (Keygen Biotech, Jiangsu, China) containing 10% fetal bovine serum (Biological Industries, Kibbutz Beit Haemek, Israel) at 37 °C and 5% CO_2_.

### Screening of baclofen concentration

SKOV3 Cells were seeded into 96-well plate at 1 × 10^4^ cells per well. When cell confluence reached 70–80%, culture media was changed to fetal bovine serum-free media. The cells were cultured for 24 h and incubated with baclofen at different concentrations (50 μmol/L, 100 μmol/L, 200 μmol/L, 400 μmol/L and 800 μmol/L) for another 24 h. After adding 10 μl CCK8 reagent, the cells were cultured for another 2 h. Eventually, absorbance was measured at 450 nm on a microplate reader (RT-6100, Rayto, USA). Cell viability was calculated accordingly.

### Experimental grouping

Cells were divided into four groups: Control, 100 μmol/L, 200 μmol/L and 300 μmol/L. For 100 μmol/L group, 200 μmol/L group and 300 μmol/L group, cells were incubated with baclofen at 100 μmol/L, 200 μmol/L and 300 μmol/L, respectively, for 24 h.

### Cell viability

IOSE80 cells and SKOV3 cells were seeded into 96-well plate at 1 × 10^4^ cells per well. When cell confluence reached 70–80%, the culture media was replaced by fetal bovine serum-free media. The cells were cultured for 24 h and then incubated with baclofen for 24 h according to the above experimental grouping. Finally, the cells were examined by CCK8 assay as indicated above.

### Cell apoptosis

IOSE80 cells and SKOV3 cells were incubated with baclofen for 24 h according to the above experimental grouping and then treated with Annexin V-FITC/PI apoptosis kit according to the manufacturer’s manual. In brief, 1 × 10^6^–3 × 10^6^ cells were collected and resuspended in 300 μL 1 × binding buffer. Cell suspension was then mixed with 3 μL Annexin V-FITC and 5 μL PI at room temperature for 10 min in the dark. After adding 200 μL 1 × binding buffer, the cells were examined immediately using a flow cytometer (NovoCyte 2060R, Acea Biosciences, China).

### Cell colony formation

SKOV3 cells were exposed to baclofen according to the above experimental grouping. The cells were then collected and seeded into 6-well plate at 300 cells per well. After culturing for 10 days, the cells were fixed in 4% paraformaldehyde for 15 min, washed three times with phosphate buffer saline (PBS), stained in 0.1% crystal violet for 45 min, washed three times with PBS again and microscopically examined.

### Cell migration

SKOV3 cells were exposed to baclofen according to the above experimental grouping. The cells were collected and seeded into 24-well plate. When cell confluence reached 90%, a scratch was made using a 10 μl pipette tip across the cell monolayer. Subsequently, the cells were washed three times with PBS. Fetal bovine serum-free media was added and the scratch was microscopically examined. After culturing for 24 h, the cells were visualized again using a microscope.

### Cell invasion

Matrigel was coated onto the membranelle of transwell inserts and cultured at 37 °C. SKOV3 cells were exposed to baclofen according to the above experimental grouping, collected and resuspended in fetal bovine serum-free media. Cell concentrations were adjusted to 1 × 10^5^ cells per ml. Cell suspension (300 μl) and complete media (500 μl) were added into upper and lower chambers, respectively. Transwell inserts were cultured for 24 h. The cells were washed with PBS for 5 min and stained in 0.1% crystal violet for 60 min. The cells in the upper chamber were removed using cotton swabs. The cells in the lower chamber were examined microscopically and counted.

### Expression of E-cadherin, N-cadherin and GABAB1 determined by RT-PCR

SKOV3 cells were exposed to baclofen according to the above experimental grouping. Total RNA was extracted using Trizon reagent and Ultrapure RNA extraction kit according to the manufacturer’s instructions. Reversed transcription of RNA to cDNA was performed using HiFiScript cDNA synthesis kit according to the manufacturer’s instruction. Primers were shown in Table 1 and added into a 25 μl PCR system which was composed of 1 μl cDNA/DNA, 1 μl forward primer, 1 μl reverse primer, 12.5 μl ULtraSYBR Mixture and 9.5 μl RNase free dH_2_O). Reaction parameters included pre-denaturation for 10 min at 95 °C, denaturation for 10 s at 95 °C, annealing for 30 s at 50 °C, elongation for 30 s at 72 °C, and 40 circles. Analysis parameters of dissociation curve included 15 s at 95 °C, 1 min at 50 °C, 15 s at 95 °C, 15 s at 50 °C, 15 s at 50 °C, and measured stepwise from 95 °C, every 0.5 °C. Finally, PCR product was examined on a RT-PCR machine (CFX Connect, Bio-Rad, USA). GAPDH served as an internal control.

**Table 1:** Primers for RT-PCR

Gene	Primer (5′-3′)	Length of primer (bp)	Length of product (bp)
E-cadherin	For: CTCACATTTCCCAACTCCTCT	21	234
	Rev: TGTCACCTTCAGCCATCCT	19	
N-cadherin	For: GCTTATCCTTGTGCTGATGTTT	22	142
	Rev: GTCTTCTTCTCCTCCACCTTCT	22	
GABAB1	For: GTGAATAGCCGCAGGGACA	19	215
	Rev: CTGGAGCCATAGGAAAGCA	19	
GAPDH	For: GAAGGTCGGAGTCAACGGAT	20	224
	Rev: CCTGGAAGATGGTGATGGG	19	

### Expression of E-cadherin, N-cadherin and GABAB1 determined by Western blot

SKOV3 cells were exposed to baclofen according to the above experimental grouping and lysed in RIPA buffer for 30 min. Cell lysate was centrifuged at 12000 rpm and 4 °C for 10 min. The supernatant was collected carefully to acquire total protein. Protein concentration was examined using a BCA kit. Subsequently, the proteins were denatured and loaded to conduct SDS-PAGE electrophoresis for 1–2 h. The proteins were transferred to membranes by a wet method for 30–90 min. The membranes were incubated in primary antibody buffer overnight at 4 °C, washed, and incubated in secondary antibody buffer for 1–2 h at room temperature. After adding chemiluminescence solution, the membranes were evaluated on a gel imaging system (ChemiDoc XRS+, Bio-Rad, USA). Relative amounts of protein per band were measured with Image Lab 5.2 software (Bio-Rad, USA).

### Statistical analysis

Every experiment was repeated five times. SPSS 19.0 software was used to carry out statistical analysis which was based on analysis of variance (ANOVA) followed by a post hoc test. Difference was considered to be significant at *P* < 0.05.

## Results

### Screening of baclofen concentration

The viability of SKOV3 cells after incubation with different concentrations of baclofen (50 μmol/L, 100 μmol/L, 200 μmol/L, 400 μmol/L and 800 μmol/L) was shown in Fig. 1a. When the baclofen concentration reached 200 μmol/L, the cell viability decreased significantly compared with the control (*P* < 0.05). Cell viability decreased significantly with increasing concentration of baclofen (*P* < 0.05), but 400 μmol/L and 800 μmol/L baclofen caused similar cell viability. Therefore, the following experiments were carried out at 100 μmol/L, 200 μmol/L and 300 μmol/L as low, medium and high concentrations of baclofen respectively.

**Fig. 1:** The viability of cells. **a** The viability of SKOV3 cells after incubation with different concentrations of baclofen (50 μmol/L, 100 μmol/L, 200 μmol/L, 400 μmol/L and 800 μmol/L). **b** The viability of SKOV3 cells and IOSE80 cells in various groups. Cells were incubated with baclofen (100 μmol/L, 200 μmol/L and 300 μmol/L) for 24 h. *P* < 0.05 vs. Control; ^#^*P* < 0.05 vs. 200 μmol/L

### Cell viability

The viability of SKOV3 cells and IOSE80 cells in various groups was shown in Fig. 1b. There was similar viability of SKOV3 cells between the control and 100 μmol/L groups. Compared with the control and 100 μmol/L groups, the viability of SKOV3 cells decreased sharply when 200 μmol/L and 300 μmol/L baclofen was exerted (*P* < 0.05). However, compared with the control group, there was no significant difference in the viability of IOSE80 cells when treated with 100, 200 and 300 μmol/L baclofen. It was suggested that baclofen only reduced the viability of ovarian cancer cells, but not normal ovarian cells.

### Cell apoptosis

The apoptosis of SKOV3 cells and IOSE80 cells in various groups was shown in Fig. 2. There was similar apoptosis of SKOV3 cells between the control and 100 μmol/L groups. The apoptotic rates of SKOV3 cells increased significantly with increasing concentration of baclofen (*P* < 0.05). However, compared with the control group, there was no significant difference in the apoptosis of IOSE80 cells when treated with 100, 200 and 300 μmol/L baclofen. These results suggested that baclofen only reduced the viability and enhanced the apoptosis of ovarian cancer cells, but not normal ovarian cells. Therefore, the following experiments were only performed in SKOV3 cells.

**Fig. 2:** The apoptosis of IOSE80 cells (**a**) and SKOV3 cells (**b**) in various groups. Cells were incubated with baclofen (100 μmol/L, 200 μmol/L and 300 μmol/L) for 24 h. *P* < 0.05 vs. Control; ^#^*P* < 0.05 vs. 200 μmol/L

### Cell colony formation

The colony formation of SKOV3 cells in various groups was shown in Fig. 3a. Compared with the control group, the cell numbers were reduced remarkably when 100 μmol/L, 200 μmol/L and 300 μmol/L baclofen was used (*P* < 0.05). Moreover, the cell numbers decreased significantly with increasing concentration of baclofen (*P* < 0.05).

**Fig. 3:** The colony formation (**a**), migration (**b**) and invasion (**c**) of cells. **a** The colony formation of SKOV3 cells in various groups. Cells were incubated with baclofen (100 μmol/L, 200 μmol/L and 300 μmol/L) for 24 h. **b** The cell scratches and mobility rates of SKOV3 cells in various groups. Cells were incubated with baclofen (100 μmol/L, 200 μmol/L and 300 μmol/L) for 24 h. **c** The cell numbers in the lower chamber of transwell assay in various groups. SKOV3 cells were incubated with baclofen (100 μmol/L, 200 μmol/L and 300 μmol/L) for 24 h. *P* < 0.05 vs. Control; ^#^*P* < 0.05 vs. 200 μmol/L

### Cell migration

The cell scratches and mobility rates of SKOV3 cells in various groups were shown in Fig. 3b. Compared with the control group, 100 μmol/L, 200 μmol/L and 300 μmol/L baclofen significantly reduced the cell mobility rate (*P* < 0.05). Moreover, the mobility rate decreased significantly with the increase of baclofen concentration (*P* < 0.05).

### Cell invasion

The numbers of SKOV3 cells in the lower chamber of transwell assay in various groups were shown in Fig. 3c. There were similar cell numbers between the control and 100 μmol/L groups. Compared with the control group, 200 μmol/L and 300 μmol/L baclofen significantly reduced the cell numbers in the lower chamber (*P* < 0.05). Moreover, the cell numbers in the lower chamber decreased significantly with the increase of baclofen concentration (*P* < 0.05).

### Expression of E-cadherin, N-cadherin and GABAB1

Figure 4 showed the mRNA and protein levels of E-cadherin, N-cadherin and GABAB1 in various groups which were examined by RT-PCR and western blot, respectively. Compared with the control group, the expression of E-cadherin and GABAB1 increased significantly and the expression of N-cadherin decreased significantly in 200 μmol/L and 300 μmol/L groups (*P* < 0.05). Higher concentration of baclofen induced higher expression of E-cadherin and lower expression of N-cadherin (*P* < 0.05).

**Fig. 4:** The mRNA and protein levels of E-cadherin, N-cadherin and GABAB1 in various groups which were examined by RT-PCR and western blot, respectively. SKOV3 cells were incubated with baclofen (100 μmol/L, 200 μmol/L and 300 μmol/L) for 24 h. *P* < 0.05 vs. Control; ^#^*P* < 0.05 vs. 200 μmol/L

## Discussion

It is generally believed that the development and progression of ovarian cancer are related to the activation of proto-oncogenes and inactivation of tumor suppressor genes. The proliferation, migration and EMT of tumor cells are important characteristics for the development and invasion of ovarian cancer [18]. Neurotransmitters are important proteins which widely exist in the central and peripheral nervous systems and they mediate neurophysiological activities of the body. GABA is the main neurotransmitter in the central nervous system and plays an important role in regulating the excitability of nerve cells [19]. The execution of GABA function depends on its unique receptor system. Hypofunction of GABA receptor system will cause epilepsy, spasm, anxiety, stress, sleep disorder, depression, addiction and pain, while excessive activation of GABA receptor will cause schizophrenia [20].

GABAB1 receptor is widely expressed in a variety of cancer tissues and cancer cells, which are closely related to the development of various cancers such as lung cancer, colon cancer, pancreatic cancer and liver cancer [21–24]. GABAB1 receptor plays a negative regulatory role in the migration of cancer cells and can also inhibit the development and progression of tumors [21–24]. Baclofen is a derivative of GABA, which can inhibit the release of excitatory amino acid, reduce the excitability of monosynaptic and polysynaptic reflexes in the spinal cord, and reduce the substance P release and calcium influx, thereby alleviating myotonia and painful spasm [25]. Therefore, baclofen is a specific activator of GABAB1 [26]. In this study, we revealed that the mRNA level of GABAB1 was significantly increased when the concentration of Baclofen reached 200 μmol/L and 300 μmol/L, while its protein level was significantly elevated when the baclofen concentration was 100 μmol/L, 200 μmol/L and 300 μmol/L. This agreed with a previous report [26]. These results suggested that baclofen could up-regulate the expression of GABAB1 and activate GABAB1.

Moreover, baclofen can inhibit the proliferation and migration of human hepatocellular carcinoma cells, lung cancer cells, gastrointestinal cancer, breast cancer and pancreatic ductal cancer cells [27–30]. This study also showed that the proliferation and migration of epithelial ovarian cancer cell line SKOV3 were significantly decreased and the cloning and invasive ability of SKOV3 cells were inhibited by baclofen at a certain concentration. Besides, baclofen at a certain concentration could enhance the apoptosis of SKOV3 cells. These results might indicate that baclofen activated GABAB1 receptor, consequently inhibiting the proliferation, cloning, migration and invasion of ovarian cancer cells and promoting the apoptosis of ovarian cancer cells.

EMT refers to the process of epithelial cells transforming into mesenchymal cells phenotype under certain conditions. Decrease of intercellular adhesion force, disappearance of the cells polarity, change of the cytoskeleton, enhancement of the ability of epithelial cells to deform, migrate and move, loss of the epithelial markers and acquirement of interstitial markers are found during this process [31]. Different types of EMT play different roles in different biological processes such as fertilized egg implantation, embryogenesis, organ development, tissue regeneration, fibrosis of epithelial tissues, invasion and metastasis of tumors [32]. EMT significantly affects the development and progression of tumors [33]. N-cadherin and E-cadherin are the focused genes in the investigation of EMT. E-cadherin is an important molecule of intercellular junction. The expression of E-cadherin is down-regulated during the EMT process, resulting in the decrease of intercellular adhesion force, while the up-regulation of N-cadherin expression is another important marker of EMT [34]. This study showed that when ovarian cancer cells were exposed to baclofen, E-cadherin expression increased significantly and N-cadherin expression decreased significantly. It was suggested that baclofen could inhibit the EMT of ovarian cancer cells.

Evaluating the influence of Baclofen incubation at different times on the SKOV3 cell line can enhance the rigor of this study. The time point of 24 h in this study was selected according to a previous report that Zhang et al. examined the role of GABA signaling molecule in breast cancer metastasis based on 24 h treatment time of baclofen [29]. Moreover, in this study, the inhibition rate of 400 μmol/L baclofen on cell proliferation exceeded 50% at 24 h, so the 24 h treatment time was chosen and no other time points were evaluated. GABAB1 and GABAB2 are the two most common subtypes of GABA B receptors and are often studied together. For example, we previously revealed that Pinocembrin inhibited the proliferation and migration of ovarian cancer cells and promoted their apoptosis by down-regulating the mRNA levels of GABAB1 and GABAB2 [35]. However, another study reported that the expression of GABAB1 in SKOV3 cells was higher than that of GABAB2, indicating that GABAB1 might be more active in SKOV3 cells [36]. Therefore, GABAB1 receptor was examined in this study. Nevertheless, the absence of GABAB2 receptor analysis was also a shortcoming of this study. In our further in-depth study, we would conduct necessary analysis of GABAB2. More cell lines can better prove the effect of baclofen on ovarian cancer cells, but SKOV3 is a commonly used cell line for studying ovarian adenocarcinoma. Paramee et al. only used SKOV3 cells to investigate the effect of Kaempferia parviflora on ovarian cancer and it was concluded that Kaempferia parviflora inhibited the proliferation, migration and invasion and induced apoptosis of ovarian cancer cells [37]. Zhao et al. also only chose SKOV3 cells to explore the combination therapies of dihydroartemisinin and curcumin for ovarian cancer [38]. Moreover, we had previously proved that Pinocembrin could down-regulate the mRNA levels of N-cadherin and GABAB receptor in SKOV3 cells and thereby inhibit the proliferation and migration of ovarian cancer cells [35]. Nevertheless, the absence of more ovarian cancer cell lines was a limitation of this study. We would conduct a further in-depth investigation in more ovarian cancer cell lines and animal model.

## Conclusion

Baclofen inhibited the proliferation, cloning, migration, invasion and EMT of ovarian cancer cells by activating GABAB1 receptor. This might contribute a lot to clarify the role and possible mechanism of GABAB1 receptor in ovarian cancer and might provide a theoretical basis for the further development of anti-cancer drugs coupled with GABAB1 receptor.

## Data Availability

All data generated or analysed during this study are included in this published article.

## Abbreviations

ANOVA: Analysis of variance
EMT: Epithelial-mesenchymal transition
FITC: Fluorescein isothiocyanate
GABA: γ-aminobutyric acid
GAPDH: Glyceraldehyde-3-phosphate dehydrogenase
GPCR: G protein-coupled receptor
PBS: Phosphate buffer saline
PI: Propidium iodide
